# Development and Evaluation of BLE-Based Room-Level Localization to Improve Hand Hygiene Performance Estimation

**DOI:** 10.1155/2023/4258362

**Published:** 2023-01-31

**Authors:** Kimia Hadian, Geoff Fernie, Atena Roshan Fekr

**Affiliations:** ^1^The KITE Research Institute, Toronto Rehabilitation Institute, University Health Network, Toronto, Ontario, Canada; ^2^Institute of Biomedical Engineering, University of Toronto, Toronto, Ontario, Canada; ^3^Department of Surgery, University of Toronto, Toronto, Ontario, Canada

## Abstract

Hand hygiene is one of the most effective ways to prevent infection transmission. However, current electronic monitoring systems are not able to identify adherence to all hand hygiene (HH) guidelines. Location information can play a major role in enhancing HH monitoring resolution. This paper proposes a BLE-based solution to localize healthcare workers inside the patient room. Localization accuracy was evaluated using one to four beacons in a binary (entrance/proximal patient zone) or multiclass (entrance/sink/right side of the bed/left side of the bed) proximity-based positioning problem. Dynamic fingerprints were collected from nine different subjects performing 30 common nursing activities. Extremely randomized trees algorithm achieved the best accuracies of 81% and 71% in the binary and multiclass classifications, respectively. The proposed method can be further used as a proxy for caregiving activity recognition to improve the risk of infection transmission in healthcare settings.

## 1. Introduction

Evidence from both the SARS and COVID-19 pandemics shows that improving hand hygiene (HH) is one of the most effective ways to prevent infections [1–5]. The Ministry of Health and Long-Term Care guidelines in Ontario, Canada, recommended that HH should be performed in 4 moments or opportunities: (1) before an initial patient or patient environment contact, (2) before performing aseptic procedures, (3) after body fluid exposure risk, and (4) after contact with a patient or patient environment [6]. HH monitoring is critical in healthcare settings where both patients and healthcare workers are at high risk of hospital-acquired infections (HAIs). Currently, the gold standard for monitoring HH is direct observation, i.e., using a trained observer to determine the adherence to HH protocols among staff. This is the only method that can identify adherence to all four moments of HH [7]. However, it is not only time-consuming and expensive, but it also fails to capture more than 97% of HH opportunities and suffers from an overestimation of performance of between 200 and 300% [7–9].

Electronic monitoring systems have been introduced to provide an accurate estimation of HH performance by detecting more opportunities without affecting healthcare workers' workflow. Although these systems provide additional valuable information regarding healthcare workers' HH adherence, they are still not able to correctly identify all 4 HH moments. The location of the healthcare worker inside the patient room can help in quantifying the exposure risk to infection for both the patients and the caregivers [10]. In general, electronic monitoring systems with some level of position-sensing capabilities can be divided into two groups. The first group localizes the healthcare worker by monitoring their entrance to the room [11–13] while the second group identifies the proximity of the healthcare worker to the patient's bed by solely monitoring a predefined zone around the bed [14–18]. While both types of systems are unable to identify moments 2 and 3, systems with room entrance monitoring may also overestimate the number of moments 1 and 4. For example, if healthcare workers enter a room and verbally check on the patient without touching the patient or the environment, they are not required to perform HH according to the protocols. However, the current systems consider this as HH moment 1 and will count this as a missed HH action. The solution is not simply to move the boundary from the door entrance to closer to the patient since mobility aids and other equipment are often scattered across the room and since if the electronic system is to be used to prompt HH, the reminder is likely to be issued when the caregiver is so close that she/he is already committed to contacting the patient or patient's proximal environment.

Incorporating localization solutions with high resolution inside the patient room can combine the benefits of both types of systems and lead to better identification of HH moments. The goal of this paper is to evaluate the performance of Bluetooth Low Energy (BLE) beacons for in-room positioning. The contribution of this work is twofold: (1) this work introduces a new era in HH monitoring by proposing multizone localization inside the patient room and (2) the proposed infrastructure for BLE module placement can be generalized to different room layouts in hospitals.

The rest of the paper is organized as follows. First, we overview the related technologies and methods used in indoor localization and review the application of indoor navigation in healthcare settings. Next, the proposed experimental setup, segmentation, feature extraction, feature selection, and classification methods are discussed. Finally, the experimental results are presented.

## 2. Related Work

While Global Positioning Systems (GPSs) provide a relatively accurate and reliable estimation of location in outdoor environments, they are not suitable for applications for indoor positioning because of a lack of signal coverage. Despite extensive research in the field of indoor positioning, no technology has yet produced similar results to what GPS offers for outdoor positioning with a comparable cost and accuracy [19]. In this section, we have reviewed different studies on indoor navigation with more focus on systems used in healthcare settings. Generally, the indoor positioning literature can be categorized by the type of technologies and the methods they use [20–25] as follows.

### 2.1. Indoor Localization Technologies

There are several technologies used in indoor localization such as inertial measurement units (IMUs), magnetic-based technology, infrared, visible light communication (VLC), ultra-wideband (UWB), Wi-Fi, radio frequency identification (RFID), and Bluetooth [22]. Typically, in systems that utilize electromagnetic waves, the frequency of the signals influences their characteristics such as wall penetration, resistance to interference, and coverage. These technologies are often used in combination with each other to achieve the best performance.

#### 2.1.1. Pedestrian Dead Reckoning (PDR)

The pedestrian dead reckoning methods use IMUs. The displacement is usually calculated by estimating the number of steps, step length, and heading direction. In this method, the initial location and orientation of the user should be input into the algorithm. Unfortunately, the accumulated errors in the displacement and heading estimation over time make the system unreliable [26].

#### 2.1.2. Magnetic-Based Technologies

Magnetic-based technologies usually measure the disturbances that occur to Earth's magnetic field due to building structures. Initially, magnetic maps are created using magnetometers in each area of the building. The location is estimated by comparing the measured values to the magnetic map. Magnetic fields are highly affected by the environment which can negatively affect the performance of these systems [22].

#### 2.1.3. Infrared

Unlike radio frequency-based technologies, infrared systems are used for their simplicity and immunity to interference. These systems usually consist of infrared transmitters which emit unique codes to the receivers in their line of sight. These systems are suitable for room-level localization; however, their performance can be adversely affected in different lighting conditions [22]. Time of flight sensors use infrared light (lasers invisible to human eyes) to determine depth information. This type of sensor has been also used to study human motions and detect steps in a wearable design [27]. However, these sensors have a limited field of view which limits them for indoor localization.

#### 2.1.4. Visible Light Communication (VLC)

In this method, data are transmitted by turning a source of visible light on and off in predefined patterns, rapidly. The flickers are usually fast enough that they cannot be perceived by human eyes. The message encoded in light modulations is generally received by a photodiode or an image sensor (e.g., a camera). The mean accuracy value reported by VLC-based systems is measured in centimetres; however, there exist challenges to using this technology such as emitter time synchronization and robustness to sunlight [25].

#### 2.1.5. Wi-Fi

Wi-Fi-based systems are popular in localization since large buildings already incorporate several Wi-Fi access points to provide coverage in different areas of the building. Furthermore, most of the current smartphones and other portable devices have built-in Wi-Fi capabilities which can reduce the need for additional infrastructure. This method also covers a wide area which can range up to 100 m–1 km [22]. However, since the existing Wi-Fi networks are originally used for communication, new processing techniques should be proposed to use this information for indoor localization [21]. Wi-Fi-based systems might also suffer from interference in their broadcasting band [28].

#### 2.1.6. Bluetooth Low Energy (BLE)

BLE systems offer cost-effectiveness, secure transmission, and power efficiency. The range offered by BLE devices is up to 100 m and they are used for localization in relatively smaller areas [22]. Fingerprinting is the most widely used method to increase accuracy in the implementation of localization in buildings [20]. Beacons are commonly used for proximity-based applications in which an action will be triggered once the user is within a specific proximity range of the beacon [21].

#### 2.1.7. Ultra-Wide Band (UWB)

Ultra-wide band refers to signals with a large bandwidth (more than 500 MHz) that emit precisely timed short pulses [24]. UWB generally has low power consumption, high-speed communication, and high time resolution and is usually resistant to interference. Although UWB-based systems provide one of the best accuracies (up to a few cm) among the localization technologies, their performance is associated with a high cost and requires additional infrastructure.

#### 2.1.8. Radio Frequency Identification (RFID)

RFID systems usually consist of RFID tags or transponders representing information and a reader that can read the data from these tags. There are three main methods of communication (coupling) between the components of an RFID system: inductive, capacitive, and backscatter. The complexity, range, and cost of the systems are influenced by their coupling methods. RFID tags are categorized based on their power supply. Passive tags do not have an embedded power source and use the power in the reader's signal. Passive RFIDs are usually cost and size-efficient but cover a limited range of up to 10 m [22]. Active tags have an onboard power source and have a significantly greater range of up to 1 km. Active RFIDs are usually used in real-time localization systems but still cannot achieve submeter accuracy [21].

#### 2.1.9. Sound-Based Technologies

These systems utilize ultrasound or audible sounds for localization purposes. Some sound-based systems can use microphones embedded in smartphones to capture modulated acoustic signals. Other sound-based systems can take advantage of the principles related to phase and frequency shifts or the speed of the acoustic waves to calculate the distance between the transmitter and the receiver. Although sound-based systems can provide accuracy in the range of centimetres, they suffer from variations in the environment such as humidity or temperature and they require high cost as well as additional infrastructure [21].

### 2.2. Indoor Localization Methods

There have been different indoor positioning techniques reported in the literature [23]. Liu et al. categorized the localization techniques into three main groups: triangulation, scene analysis (fingerprinting), and proximity [29]. Triangulation combines measurements in time (angulation) or distance (lateration) using geometric properties of triangles. Lateration methods can be further classified into five groups based on their use of measurement, namely, time of arrival (ToA), time difference of arrival (TDoA), round time of flight (RToF), phase of arrival (PoA), and received signal strength (RSS).

The distance between the signal transmitter and receiver can be measured using propagation time. In this method, which is called ToA or ToF, the transmitters and receivers are required to be precisely synchronized and the emitted signals need to have a timestamp. The distance between the receiver and transmitter is calculated by multiplying the time required for the signal to travel from the transmitter to the receiver at the speed of light. Another approach is measuring the time difference between the received signal at multiple measuring units, i.e., TDoA, and converting it into distance. Since this method conventionally uses correlation techniques between the received signals, there is no need for synchronization between the transmitter and receivers; however, the receivers should still be precisely synchronized. In order to create a more moderate synchronization requirement, RToF can be used. In this method, the time of flight of a signal from the transmitter to the receiver and the reverse is measured. Unlike ToA methods that use multiple nodes to calculate the time difference, RToF only uses one node to record the transmitting and arrival time; therefore, it is less prone to synchronization issues [30]. Instead of time or time difference in the methods mentioned above, POA uses the phase or the phase difference in the transmitted and received signals. These methods suffer from inadequacies when there is no clear line of sight between the transmitter and the receiver. A signal attenuation model can be used to compensate for the effect of the environment.

Received signal strength (RSS) combined with an attenuation model is used to estimate the distance between the receiver and the transmitter. The parameters of this model are usually set according to the characteristics of the environment. Likewise, if the distance between two nodes is known, the distance between these nodes and the target can be calculated by determining the angles between each known node and the target. This method is called angulation or angle of arrival (AoA). This method does not need any synchronization; however, the localization errors will increase as the distance between the target and nodes increases.

Scene analysis (fingerprinting) methods consist of two steps. In the first step, the offline phase, several signals and features are collected from an environment in different locations. In the second phase, this collected information (fingerprints) is used to predict the location of the target based on the new signals. Several models such as neural networks, support vector machines, K-nearest neighbors, and probabilistic models have been used in the literature for scene analysis. Fingerprinting is a simple method that is widely used in RF localization [25, 31]. However, this technique is not only time-consuming but also has to be updated as the environment changes. New methods incorporating crowdsourcing are being used to make this method more efficient [32, 33].

### 2.3. Indoor Localization in Healthcare Settings

Indoor localization solutions in healthcare settings can be divided into wayfinding applications for healthcare workers and patients, HH monitoring, and patient and asset tracking. The authors in [34] used Wi-Fi access points and AoA method to propose an outpatient wayfinding application. They achieved less than 2.5 m accuracy in 80% of the cases in a line of sight (LOS) environment using an algorithm for smartphones. The drawbacks of this work include the high cost of infrastructure and lower accuracy in non-LOS environments. Calderoni et al. used RFID technology and fingerprinting technique for patient tracking [35]. The collected fingerprints are first clustered into micro-areas with rooms that are in the relatively same area and then a random forest classifier is used to estimate the final location. This approach was able to estimate the correct room with an 83% accuracy. The authors in [36] combined Wi-Fi and RFID technology to compensate for the shortcomings of each technology and achieved an accuracy of less than 4 m for patient tracking. Van Haute et al. compared the performance of Wi-Fi, BLE, and Zigbee technologies using three methods in healthcare settings [37]. Their findings indicate that fingerprinting is the most accurate and robust algorithm compared to ToA and attenuation models. However, if latency, environmental robustness, installation cost, and time are of importance, other methods should be considered. They reported that the choice of technology has minimal impact on accuracy. The authors concluded that a combination of fingerprinting algorithm and Wi-Fi technology provided the highest accuracy; however, cheaper technologies such as BLE and Zigbee are better alternatives if latency, power consumption, and cost optimization are required. Another study that compared geomagnetic, Wi-Fi, and BLE technologies in a hospital environment concluded that even though the geomagnetic technology was the most accurate technology, the combination of geomagnetic and BLE yielded the best performance [38]. Localization for HH monitoring is often embedded in commercial systems. There is a wide variety of commercial location tracking systems combined with infection control use cases for healthcare settings.  Table 1 provides a summary of the systems discussed.

As mentioned above, current electronic monitoring systems are not capable of positioning the caregiver inside the room. The localization of healthcare workers inside the patient's room can enhance the current calculation of HH performance (compliance rate) as well as the new parameter called patient exposure risk (PER) introduced in [10]. The authors in [45] used a motion capture system to derive the location and orientation of the caregiver inside the room and showed that the caregiving activities are well related to their location in the nursing environment. The main goal of our study is to detect the position of the caregiver inside the room without adding cumbersome infrastructure that will hinder their workflow. This goal will be achieved by evaluating the performance of different numbers of low-cost BLE beacons in different locations of the room.

## 3. Proposed Methodology

Depending on the resources available and the required resolution, the indoor positioning problem can be approached as a binary or a multiclass classification problem. In the binary classification, the patient room is divided into two main zones: the entrance zone (Z1) and the patient zone. The goal is to identify whether the caregiver has entered the patient zone. The multiclass classification problem aims to increase the resolution of the localization by dividing the room into four zones: the entrance zone (Z1), the sink zone (Z3), the left side of the patient's bed (Z4), and the right side of the patient's bed (Z2), as shown in Figure 1. In this paper, we use BLE beacons in different locations of the room (B1–B4 in Figure 1) to localize the caregiver inside the room. Data collection took place in CareLab located at KITE Research Institute, Toronto Rehabilitation Institute, UHN. The lab simulates a typical hospital patient care room. Nine healthy participants were recruited to perform several activities including walking, standing, and a list of 29 common nursing activities listed in Table 2. The performance of the BLE localization is influenced by the line of sight and the relative speed of the transmitters and the receiver; therefore, including a wide variety of activities is required to achieve more realistic results. The protocol was approved by the University Health Network Ethics Board, and written consent was obtained from the participants.

### 3.1. Experimental Setup

BLE 4.0 beacons (Blue Charm LLC, Eugene, USA) were used to collect information about the participant's location in the room. These beacons are low-energy transmitters that broadcast small packets of data at regular customizable intervals within a short range. There are two main broadcasting protocols, iBeacon by Apple and Eddystone by Google. Despite some minute differences between the information broadcast by each protocol, both can be used on iOS and Android devices and these differences have no impact on the end-users of our system. In this study, the iBeacon communication protocol with a customized iOS application was used to collect the BLE data. The iBeacon packets contain a universally unique identifier (UUID), a major parameter, and a minor parameter. For example, beacons in the same hospital have similar UUIDs, beacons in the same unit have the same major values, and beacons in each room are specified by their minor values. These packets are received by a BLE receiver such as a smartphone (in our case an iPhone 11) when in range. Additional information such as the received signal strength indicator (RSSI), proximity, and accuracy can be obtained once a beacon is detected. The proximity value is a categorical value that reports the proximity of the receiver to the beacon based on the estimated distance. The reported values are “immediate,” “near,” “far,” and “unknown.” The “immediate” value indicates that the receiver is very close to the beacon (less than 1 m). With a clear line of sight, the “near” value represents a distance of 1–3 m between the beacon and the receiver. The “far” value indicates that the beacon can be detected but the ranging cannot be reported with confidence. Lastly, the proximity value is “unknown” if the beacon is not accurately detected. The accuracy value can be used to differentiate between the beacons with the same proximity values. The lower accuracy values indicate that the receiver is closer to that beacon [46]. In our study, 4 beacons were installed above the door (B1), on the wall opposite the door (B2), above the sink (B3), and above the bed (B4) (see Figure 1). These placements are chosen in such a way that they can be generalized to any room layout. The phone was placed in the front pocket of the participants' scrub. As depicted in Figure 1, the room was divided into four different zones: entrance, sink, right, and left side of the bed. Once the app detects a beacon, it will store the UUID, major, minor, proximity, accuracy, RSSI, and timestamp. The timestamped locations of the participants were logged by a trained observer as the true labels. In addition to the location of the beacons, the transmission power can be adjusted between three levels (−23 dB, −6 dB, and 0 dB). In our data collection, we experimentally chose 0 dB for the transmission power.

### 3.2. Data Analysis

About 26.5 hours of data (95,000 samples for each beacon) were collected for this study. Since the quality of the collected data is critical in a classification problem, we tested different parameters both in the data acquisition and the data preprocessing stages to obtain an information-rich dataset.  Figure 2 depicts the histogram of the data collected from all the beacons for different zones. As can be seen from this figure, the distribution of the RSSI and accuracy signals do not change significantly with location. This is mainly caused by the low signal-to-noise ratio and due to the fact that unlike other applications in the previous literature, our entire testing environment is as small as a 5 × 5 m^2^ room.

Recursive feature elimination (RFE) with cross-validation was used to choose the most useful feature set. RFE is performed by recursively removing features with low importance weights assigned by an external estimator [48]. As shown in Figure 3, walking is the dominant activity in our dataset in all zones. In other words, the fingerprints are mostly derived in a dynamic setting as opposed to a conventional static setting where the Bluetooth receiver does not move during the offline phase of fingerprinting. It also shows that the dataset is imbalanced towards the entrance zone with the sink class having the minimum number of samples. The extracted features were balanced using the synthetic minority oversampling technique (SMOTE) before training the model [49]. In this method, samples are synthesized using the following steps: (1) a random sample of the minority class is selected (*S*_*i*_), (2) K-nearest neighbors in the minority class with respect to this sample are identified, (3) one neighbor is chosen randomly (*S*_*nn*_), and finally (4) a synthetic sample is generated at *S*_new_ = *S*_i_ + *r*(|*Si*–*S*_*nn*_|) where *r* is a random number between 0 and 1.

An ensemble of extremely randomized trees (also known as extra trees) is then trained and tested on these samples [50]. Extra tree classifiers introduce another level of randomness to tree ensemble methods by randomly choosing the cutpoints at each node instead of finding the optimal one to diversify the trees, decrease the high variance of tree-based methods, and increase the computational efficiency. The algorithms were implemented in Python using the Scikit-learn library [51].

## 4. Experimental Results and Discussion

The training and evaluation of the models were done using leave-one-subject-out (LOSO) cross-validation to minimize the overlap between the training and validation datasets. Furthermore, the oversampling was performed only for the training set in each iteration to select the best model. F1-score, precision, and recall are used to compare different models. Precision is the ratio of correctly labeled positive instances to all the positive labeled instances by the model. Recall is the ratio of correctly labeled positive instances to all the actual positive instances. F1-score is defined as the harmonic mean of the precision and recall and is calculated as follows:

(1) $$\begin{array}{c} precision=\frac{TP}{TP+FP}\text{,} \end{array}$$

(2) $$\begin{array}{c} recall=\frac{TP}{TP+FN}\text{,} \end{array}$$

(3) $$\begin{array}{c} F1=2\times \frac{precision\times recall}{precision+recall}, \end{array}$$

TP, FP, and FN represent the number of true positives, false positives, and false negatives, respectively. These metrics can be used for evaluating binary as well as multiclass classifications. In multiclass classifications, the metrics are calculated for each class separately and the arithmetic mean of all the scores is reported as the macro-averaged score or the macro-score for the model. F1-score is especially useful when dealing with imbalanced datasets but should be used with caution since it gives equal weight to precision and recall. For example, in our binary classification, misclassifying an entrance to the patient zone is worse than incorrectly classifying an event as an entrance to the patient zone since it imposes a greater risk of infection on the patient. In other words, a high recall rate is more desirable than a high precision rate. As a result, throughout this paper, in addition to the F1-score, precision and recall rates are reported. The analysis for the binary classification (Z1 and ∼Z1) was done using only one beacon with four placements. Combinations of different beacon placements were however tested in our multiclass case (Z1-Z2-Z3-Z4).

### 4.1. Data Segmentation Analysis

We have investigated the effect of different segmentation techniques, i.e., fixed-size non-overlapping sliding windows and fixed-size overlapping sliding windows with several window sizes in binary and multiclass classifications. We tested window sizes of 3, 5, and 10 seconds with 0%, 20%, 40%, 60%, and 80% overlap values. The results are obtained using the features extracted from the accuracy and RSSI signals.

As shown in Figure 4(d), B4 (located above the bed) with non-overlapping windows of size 5 s resulted in the best F1-score of 0.84 for binary classification. The next beacon with the highest performance was located above the sink (B3) with an F1-score of 0.74, followed by B1 and B2 both with F1-scores of 0.72, all with window size = 5 s. The significant difference in performance observed from B4 compared to other beacons could be due to the fact that the participants spent most of their time close to B4. Moreover, the static fingerprints were mostly collected close to the bed and therefore closer to B4. As shown in Figure 4, the worst case F1-scores were achieved using non-overlapping 10 s windows. The reason is that in 10 s, the subjects have enough time to travel from one zone to another, leading to mislabeling the window in the majority voting method. On the other hand, 5 s windows provide enough samples for the classifier to distinguish the current zone without the participant moving to another one. Since extra tree forests are used for classification, higher overlap values lead to overfitting and therefore a decrease in the models' performance. Window size of 3 s shows the highest F1-score among all three window sizes when increasing the overlap in all cases.

Two types of fading occur during signal propagation. Large-scale fading or path loss refers to the power attenuation due to the distance between the receiver and the transmitter. Small-scale fading or multipath fading represents rapid changes in the signal's phase and amplitude that can be caused by the reflection of the waves or the movement of the transmitter or the receiver [47]. In our case, the movement of the participant, changes of orientation with respect to the beacons, and the walls and the equipment in the room created significant small-scale fading effects. In most cases, the envelope of the received signal is modelled by a Rayleigh distribution if there is no line-of-sight component and by a Rician distribution if there exists a line-of-sight component which can explain the distributions observed in Figure 2 [47]. The small-scale fading creates a high-frequency noise in our signals. Therefore, the signals are filtered using a second-order low-pass Butterworth filter with a cutoff frequency of 0.1 Hz. Next, the RSSI and accuracy signals were segmented into fixed-size overlapping and non-overlapping sliding windows. The features were extracted from these segments to train our classification model.  Table 3 shows a complete list of features used in this study.

We ran all combinations of the beacons for classifying our 4 zones. In total, 225 classifiers were tested to obtain the best placements inside the room for our multiclass classification.  Figure 5 shows the locations that resulted in the best F1-score values using 1, 2, 3, and all 4 beacons.

As expected, using 5 s non-overlapping windows with all the beacons resulted in the best F1-score of 0.67 (Figure 5(o)). Similar to the binary classification, B4 in Figure 5(d) and B1 in Figure 5(a) provided the highest and lowest F1-score with a single beacon, respectively. It was observed that the performance was dependent on both the number and the location of the beacons used. For example, B4 alone outperformed the results of the fusion of B1 and B2; however, combining B2 and B4 resulted in better performance compared to B4, separately. The gap between F1-score using different window sizes was significantly less in multiclass compared to binary classification. However, in most cases, a window size of 5 s resulted in the best performance while 10 s windows resulted in the worst case F1-score. While increasing the number of beacons from 1 to 2 and from 2 to 3 resulted in a performance increase of about 5%, increasing the number from 3 to 4 resulted only in a 2% improvement.

Figure 6 compares the F1-score, recall, and precision for distinguishing different zones as well as the macro-F1-score, macro-recall, and macro-precision when using 1, 2, 3, and all 4 beacons. The best F1-score, precision, and recall in the best models are obtained for Z1 (the entrance zone). It is important to note that the critical zones in infection control are the patient zones, i.e., Z2 and Z4 (right and left side of the patient bed) in our study. Therefore, the performances of these two zones are as critical as the overall performance. A combination of B2 and B4 (B24) shown with a yellow line in Figure 6(b) provided the best result among all 6 combinations of two beacons. B2, B3, and B4 (B234) was the best case for three beacons and finally, using all 4 (B1234) beacons provided the best performance with a macro-F1-score of 67%, as shown in Figure 6(c).

As summarized in Table 4, in all cases, a window size of 5 s and an overlap of 0% provided the best results. The reported precision and recall scores do not show a significant difference in multiclass classification.

Figure 7 represents the misclassification rates obtained from the best classifiers using one, two, three, and four beacons. In all cases, Z1 has the lowest misclassification rates. The entrance zone (Z1) is often misclassified as Z4 (left side of the bed) or Z3 (the sink). The highest misclassification rate was for Z4 (left side of the patient bed) in all cases. Increasing the number of beacons to 3 and 4 resulted in a more than 10% decrease in Z4's misclassification rate.

For binary classifications, B4 with non-overlapping windows of 5 s yielded the highest F1-score of 84%. Entrance to the patient zone was detected with 89 ± 5% accuracy. Similarly, in 76 ± 12% of the time, the model correctly labeled the events where the participants did not pass the entrance zone boundary (Figure 8). The high standard deviation in this class is mainly caused by subject 8 (Figure 8(h)). Overall, the lowest performances belonged to subjects 8 and 9 (Figures 8(h) and 8(i)). It is interesting to note that the experimental sessions for these two subjects took place on the same day. Given that the beacons, their locations, and the study setup were constant during the whole study, this could be due to the adverse effect of environmental noise. Finally, the model was more sensitive to the positive class (entrance to the patient zone) for most subjects which is desired for our application.

## 5. Limitations

In general, the signals obtained from the BLE beacons are extremely noisy and may not be suitable for localization with high resolution. Our experiments depicted in Figure 9 showed that the attenuation in the RSSI signal follows a logarithmic path loss model when the distance is less than 2 m in a line-of-sight environment. However, for distances more than 2 m, this equation does not hold. In the experiment depicted in Figure 9, two beacons were placed right next to each other in a clear line of sight, and fingerprints were collected at distances in the range of 0.5 m to 9 m with an increment of 0.5 m. At each point, the receiver was held in front of the beacon for 1 minute without any movement. When used in non-line-of-sight scenarios and with interferences from the environment, the logarithmic attenuation pattern becomes even less evident due to the large and small fading effects explained earlier. Given that the beacons were installed on the wall close to the ceiling to limit any unwanted interactions with the beacons, the distance between the receiver (the phone) and the beacons is more than 2 m in most cases. This makes accurate localization in the small patient room a challenging task.

The proposed method used in this study needs an initial phase for fingerprinting collected in each new room layout which can be time-consuming and expensive. During the study, the same device (an iPhone 11) was used as the receiver. The signals collected using different devices may slightly vary. Therefore, fingerprints should be collected using all devices that are intended to be used as a receiver.

Another limitation is that the received signals can be influenced by the number of people present in the room since the human body can absorb and cause fluctuations in the emitted signals. Another constraint was imposed by Apple. The receiver device only reported the received signals at a 1 Hz rate, which caused limitations during segmentation and feature extractions with smaller window sizes. In addition to the limitations listed above, using RF waves may cause interference with other medical devices in the hospital. Finally, the models were trained with limited data and subjects, and a larger dataset can improve the classification performance.

## 6. Conclusion

This paper proposed an adjustable indoor localization system incorporating cost-effective BLE beacons. The system is suitable for positioning the healthcare workers inside the patients' rooms to improve the existing HH monitoring systems. Depending on the resources available and the required resolution, up to four beacons can be used in the room to identify the entrance to the patient zone or the approximate location of the caregiver inside the room. Indoor localization can be used as an aid to caregiving activity recognition and HH moment detection. This can lead to a better estimation of the risk of exposure to infection for patients and healthcare workers. This work can be a foundation for increasing the localization resolution of HH monitoring systems since RSSI can be derived from most of the signals used in current systems. In the future, this can be combined with other localization techniques, such as PDR, to increase the accuracy of the system while reducing the cost and the number of beacons required.

## Figures and Tables

**Figure 1:** Beacon placements (B1–B4), room layout at CareLab, and four zones (Z1–Z4).

**Figure 2:** Distribution of RSSI received by (a) B1, (b) B2, (c) B3, and (d) B4, as well as distribution of accuracy signals received by (e) B1, (f) B2, (g) B3, and (h) B4 in all 4 zones.

**Figure 3:** The rectangular tree map that represents the dataset for each zone and each activity. The three small rectangles in Z1 represent activities 16, 24, and 29.

**Figure 4:** Effect of different window sizes and overlap values on binary classification using (a) B1, (b) B2, (c) B3, and (d) B4.

**Figure 5:** Effect of different window sizes and overlaps on multizone classification using (a) B1, (b) B2, (c) B3, (d) B4, (e) B1 and B2, (f) B1 and B3, (g) B1 and B4, (h) B2 and B3, (i) B2 and B4, (j) B3 and B4, (k) B1, B2, and B3, (l) B1, B2, and B4, (m) B1, B3, and B4, (n) B2, B3, and B4, and (o) B1, B2, B3, and B4.

**Figure 6:** F1-scores with (a) one beacon, (b) two beacons, and (c) three and four beacons, recall with (d) one beacon, (e) two beacons, and (f) three and four beacons, and precision with (g) one beacon, (h) two beacons, and (i) three and four beacons. Bxyzw represents the results when using beacons *x y*, *z*, and *w*.

**Figure 7:** Misclassification rates for the best models using (a) one beacon, (b) two beacons, (c) three beacons, and (d) four beacons. (e) Room layout and four zones. The colors in the map correspond to the colors specified for each zone in the bar graphs.

**Figure 8:** Confusion matrices for the best model for binary classification; true/false labels represent cases where the participant did/did not cross the entrance threshold. Each confusion matrix (a–i) corresponds to an individual subject (1–9).

**Figure 9:** Comparison of RSSI between two beacons at different distances.

**Table 1:** Commercial location tracking systems used in healthcare environments (WSN: wireless sensor network, RFID: radio frequency identification, IR: infrared, and BLE: Bluetooth Low Energy).

Device	Technology	Application	Resolution
Polgreen [13]	WSN	HH monitoring	Room level
General Sensing, MedSense Clear [15, 17]	RFID	HH monitoring	Zone level
EcoLab [14]	WSN	HH monitoring	Zone level
Hygienic Echo-Buddy Badge [11, 39]	IR	HH monitoring	Room level
Sani Nudge [16, 18]	BLE	HH monitoring	Zone level
Sonitor [40]	Ultrasound	Asset management, patient flow, staff workflow, HH monitoring	Room level
MidMark [41]	BLE, IR, Wi-Fi	Patient flow, asset management, contact tracing	Zone level
CenTrak [42]	IR, RFID, Wi-Fi	Asset management, staff workflow, HH monitoring	Room level
Stanley Healthcare-AeroScout [43]	Wi-Fi, ultrasound	Asset management, patient flow, staff workflow, HH monitoring	Room level
GE Healthcare-Encompass [44]	BLE	Asset management	Room level

**Table 2:** Activity descriptions and their corresponding codes.

Code	Activity description
1	Walking
2	Turning the light on or off
3	Opening the door
4	Closing the door
5	Opening the curtain around the bed
6	Closing the curtain around the bed
7	Moving an object on the bedside table
8	Using an ABHR dispenser
9	Moving the overbed table to the side
10	Moving the overbed table towards the bed
11	Pulling the bedside rails up
12	Pushing the bedside rails down
13	Adjusting the bed settings
14	Touching one's face or hair
15	Touching one's phone
16	Replacing an IV bag
17	Turning the patient on the bed
18	Putting a bedpan under the patient
19	Assisting the patient to sit on the side of the bed
20	Assisting the patient in walking without any walking aids
21	Assisting the patient in moving with a walker
22	Assisting the patient in moving from the side of the bed to a wheelchair
23	Moving a wheelchair
24	Assisting the patient to put on a coat
25	Assisting the patient to take off a coat
26	Using a stethoscope
27	Measuring patient's blood pressure using a digital sphygmomanometer
28	Measuring patient's pulse
29	Measuring patient's temperature using an ear thermometer
30	Measuring patient's oxygen saturation level with a pulse oximeter

**Table 3:** List of features derived from accuracy and RSSI windows (“*n*” denoted the number of samples in each window).

Feature	Description
Mean	*μ*=1/*n*∑_*i*=1_^*n*^*s*_*i*_
Standard deviation	$\sigma =\sqrt{1/n\sum_{i=1}^{n}{\left(s_{i}-\mu \right)}^{2}}$
Minimum	min(*s*_1_, *s*_2_,…, *s*_*n*_)
Maximum	max(*s*_1_, *s*_2_,…, *s*_*n*_)
Mean absolute deviation	1/*n*∑_*i*=1_^*n*^|*s*_*i*_ − *μ*|
Peak-to-peak amplitude	max(*s*) − min(*s*)
Median	median(*s*_1_, *s*_2_,…, *s*_*n*_)
25^th^ percentile	*s*_*j*_, *j*=*n*/4 where values of the window are ranked in ascending order
75^th^ percentile	*s*_*j*_, *j*=3*n*/4 where values of the window are ranked in ascending order
Interquartile range	*q*_3_(*s*) − *q*_1_(*s*)
Root mean square	$\sqrt{1/n\sum_{i=1}^{n}s_{i}^{2}}$
Power	∑_*i*=1_^*n*^*s*_*i*_^2^
Kurtosis	1/*nσ*^4^∑_*i*=1_^*n*^(*s*_*i*_ − *μ*)^4^
Skewness	1/*nσ*^3^∑_*i*=1_^*n*^(*s*_*i*_ − *μ*)^3^
Peak intensity	The number of signal peaks within a certain window
Mean of first n peaks	Mean of the largest *n* peaks in the window

**Table 4:** Best models using different number of beacons.

Beacon #	Classification	Window size (s)	Overlap (%)	F1-score	Accuracy	Recall	Precision
B4	Binary	5	0	0.84	0.81	0.88	0.80
B4	Multiclass	5	0	0.56	0.60	0.57	0.57
B24	Multiclass	5	0	0.61	0.65	0.62	0.61
B234	Multiclass	5	0	0.65	0.69	0.66	0.65
B1234	Multiclass	5	0	0.67	0.71	0.67	0.68

## Data Availability

Access to data is restricted due to University Health Network's Research Ethics Board regulations.
